The article "The Level of HbA1c Evaluates the Extent of Coronary Atherosclerosis Lesions and the Prognosis in Diabetes with Acute Coronary Syndrome" was retracted in 2023. Reason: concerns about the peer review.

# The Level of HbA1c Evaluates the Extent of Coronary Atherosclerosis Lesions and the Prognosis in Diabetes with Acute Coronary Syndrome

**DOI:** 10.1155/2022/7796809

**Published:** 2022-07-22

**Authors:** Shaodong Xu, Birong Zhou, Bingfeng Zhou, Jianfa Zheng, Qinghe Xu, Bing Wang, Minmin Fu, Ying Meng

**Affiliations:** ^1^Department of Cardiology, The First Affiliated Hospital of Anhui Medical University, Hefei, 230031 Anhui, China; ^2^Department of Cardiology, The Third Affiliated Hospital of Anhui Medical University, Hefei, 230001 Anhui, China

## Abstract

**Background:**

The level of HbA1c can reflect the average level of blood glucose over 3 months, which is the gold standard indicator for monitoring blood glucose. The relationship between the level of HbA1c and the extent of coronary atherosclerosis lesions or the prognosis in diabetes with acute coronary syndrome (ACS) remains poorly understood.

**Aims:**

To explore whether the level of HbA1c can evaluate the extent of coronary atherosclerosis lesions or the prognosis in diabetes with acute coronary syndrome (ACS) using the SYNTAX score, the Global Registry of Acute Coronary Events (GRACE) score, left ventricular function (LVEF), left ventricular end-diastolic volume (LVEDV), and major adverse cardiac events (MACEs) in the hospital and 12 months after discharge.

**Methods:**

This study was a prospective, randomized, open-label, and parallel group study. Patients with diabetes with ACS were recruited into this study indiscriminately, and all the participants were divided into two groups according to the level of HbA1c: HbA1c level ≤ 7%group and HbA1c level > 7%group. The followings were used as the evaluation indicators: SYNTAX score, GRACE score, LVEF, LVEDV, and MACEs in hospital and 12 months after discharge.

**Results:**

A total of 233 patients with diabetes and ACS were enrolled and assigned to two groups according to their level of HbA1c: the HbA1c ≤ 7%group (*n* = 92) and the HbA1c > 7%group (*n* = 141). The results showed that the proportion of STEMI was higher in the HbA1c ≤7% group (*p* < 0.05), while the proportion of NSTEMI has not significantly higher in the HbA1c >7% group (*p* > 0.05). Regression analysis indicated that HbA1c level was significantly positively correlated with GRACE score (*r* = 0.156, *F* = 5.784, *p* = 0.017, *n* = 233) and SYNTAX score (*r* = 0.237, *F* = 13.788, *p* < 0.001, *n* = 233), and there were no statistically significant differences in LVEDV and LVEF between the two groups (*p* > 0.05). The total MACEs rate showed no significant difference between the two groups during hospitalization (*p* > 0.05) but showed significant differences at 12 months after discharge (*p* < 0.05).

The article "The Level of HbA1c Evaluates the Extent of Coronary Atherosclerosis Lesions and the Prognosis in Diabetes with Acute Coronary Syndrome" was retracted in 2023. Reason: concerns about the peer review.

**Conclusions:**

This study shows that HbA1c level was positively correlated with the extent of coronary atherosclerosis lesions and the prognosis in diabetes with ACS. The higher the HbA1c level is, the more severe the coronary atherosclerotic lesion and the worse the prognosis in diabetes with ACS are.

## 1. Introduction

The International Diabetes Federation (IDF) estimated that there are 463 million diabetic patients worldwide, and this number will reach 578 million by 2030 [1]. The level of HbA1c can reflect the average level of blood glucose over 3 months, which is the gold standard indicator for monitoring blood glucose. The relationship between the level of HbA1c and the extent of coronary atherosclerosis lesions or the prognosis in diabetes with acute coronary syndrome (ACS) remains poorly understood. In diabetes, compared with the absence of diabetes, the relative risk of cardiovascular diseases (CVDs) is between 1.6 and 2.6 [2, 3], with coronary artery disease (CAD) making up approximately 21% of this risk [4], and the risk of early death and major adverse cardiovascular events (MACEs) is significantly increased in acute coronary syndrome (ACS) patients [5].

A new research hotspot is how to find a rapid and simple method to evaluate the extent of coronary atherosclerotic lesions, predict their prognosis, provide timely guidance for diagnosis and treatment, and improve the prognosis of diabetes, especially when complicated with ACS, which includes unstable angina pectoris (UA), non-ST-segment-elevation myocardial infarction (NSTEMI), and ST-segment-elevation myocardial infarction (STEMI).

The level of blood glucose is related to the occurrence and progression of CAD, and blood glucose variability is related to coronary plaque vulnerability in ACS [6], but there are many factors influencing blood glucose. HbA1c level, which has good stability, can reflect the average level of blood glucose over the preceding 3 months and is the gold standard indicator for monitoring blood glucose. Studies have shown that HbA1c level is an independent risk factor for CAD [7]. A higher HbA1c level in patients undergoing coronary angiography is associated with an increased prevalence of comorbidities [8]. Higher HbA1c level is associated with higher coronary and peripheral atherosclerotic burden in nondiabetic patients [9].

However, few studies have explored the relationship between HbA1c level and the extent of coronary atherosclerosis lesions or the prognosis in diabetes with ACS.

The purpose of this research was to study whether the level of HbA1c can evaluate the extent of coronary atherosclerosis lesions or the prognosis in diabetes with ACS using the SYNTAX score, the Global Registry of Acute Coronary Events (GRACE) score, left ventricular function (LVEF), left ventricular end-diastolic volume (LVEDV), and MACEs in the hospital and 12 months after discharge.

The article "The Level of HbA1c Evaluates the Extent of Coronary Atherosclerosis Lesions and the Prognosis in Diabetes with Acute Coronary Syndrome" was retracted in 2023. Reason: concerns about the peer review.

## 2. Methods

### 2.1. Study Population

The study was a prospective, randomized, open-label, and parallel-group study. Patients with diabetes with ACS were hospitalized in the cardiovascular department of our hospital from January 2019 to December 2020. All patients who came to our hospital emergency department or outpatient department were diagnosed with diabetes complicated with ACS and did not meet the exclusion criteria and were recruited into this study indiscriminately. Standard treatment for diabetes and ACS was given during hospitalization and after discharge. All the participants underwent percutaneous coronary angiography and percutaneous coronary intervention when necessary. The exclusion criteria were those diseases that can affect our test indicators, interfere with our results such as previous coronary artery bypass grafting, valvular heart disease, myocarditis, cardiomyopathy, severe liver, kidney, lung, and other important organ diseases such as malignant cancer, severe anemia, hyperthyroidism, rheumatic diseases, and autoimmune diseases. This study was approved by the hospital ethics committee, and all the participants signed informed consent.

### 2.2. Grouping

This study was double-blind, the results of HbA1c level after admission were sealed, neither the patient nor the researcher knew the results of HbA1c level; so, they did not know the grouping of patients. The HbA1c level and grouping of patients were known only when the final statistical results were known. In the end, the participants were divided into two groups according to the level of HbA1c: HbA1c ≤ 7% group (*n* = 92) and HbA1c > 7%group (*n* = 141).

### 2.3. Clinical Characteristics of the Patients

The general data of all the participants were recorded: sex, age, weight, height, smoking history, drinking history, past history, current history, family history, type of ACS, routine examination of blood glucose, blood lipid analysis, liver and kidney function, urinalysis, and routine blood and stool tests. The following indicators were noted at admission: heart rate, arterial systolic pressure, creatinine, ST segment change of ECG, Killip classification of cardiac function, cardiac arrest at admission,+ and elevation of cardiac markers.

### 2.4. Measurement of the HbA1c Level

Two milliliters of venous blood were collected from all the participants, anticoagulated in an EDTA tube, and sent to the laboratory of our hospital to test the level of HbA1c by using ion-exchange high-performance liquid chromatography with a Bio-Rad Variant Hemoglobin Testing System (Bio-Rad Laboratories, USA).

The article "The Level of HbA1c Evaluates the Extent of Coronary Atherosclerosis Lesions and the Prognosis in Diabetes with Acute Coronary Syndrome" was retracted in 2023. Reason: concerns about the peer review.

### 2.5. Coronary Angiography

All the participants underwent percutaneous coronary angiography and percutaneous coronary intervention using digital subtraction angiography when necessary during hospitalization. Percutaneous coronary angiography was performed using radial, brachial, or femoral artery puncture, and the catheter was sent to the left and right coronary artery ostium. The results of percutaneous coronary angiography were recorded; stenosis of the CAD was defined as the degree of stenosis of the left and/or right coronary arteries and their main branches ≥ 50%.

### 2.6. SYNTAX Score

The 16-segment method of the coronary artery tree was used to score the lesions with a diameter ≥ 1.5 mm and a stenosis degree ≥ 50%, combined with the dominant distribution, lesion location, stenosis degree, and pathological characteristics of the coronary artery. Two senior physicians who performed the percutaneous coronary intervention systematically analyzed the results and used the online SYNTAX scoring system (http://www.syntaxscore.com) according to the location, stenosis, bifurcation, calcification, and diffusion. Each lesion was graded one by one, and then the score was added to obtain the patient's SYNTAX score [10].

### 2.7. GRACE Score

According to the Global Acute Coronary Event registration (GRACE) scoring standard, the GRACE score was calculated based on the following indicators at admission: age, heart rate, systolic pressure, creatinine, ST segment change displayed by ECG, Killip grade of cardiac function, cardiac arrest, and elevation of cardiac markers [11].

### 2.8. Left Ventricular Function

All the participants were examined by cardiac Doppler ultrasound, which recorded the following indicators: left ventricular ejection fraction (LVEF), left ventricular end-diastolic volume (LVEDV), and other indicators.

### 2.9. MACEs

MACEs were recorded in the hospital and at 12 months after discharge for all the participants. They included death, recurrence of ACS, ventricular arrhythmia/fibrillation, and revascularization.

### 2.10. Statistical Analysis

Data were processed using SPSS Statistics 22.0, and the numerical variables are expressed as mean ± standard deviation. All the statistical indicators were checked for normality and homogeneity of variances, and then measurement data were compared by the independent samples one sided *t*-test. Enumeration data were treated with the Pearson chi-square test, except that one side Fisher's exact test was used when the theoretical frequency was less than 5 or the total frequency was less than 40. The linear regression analysis method was adopted to analyze the correlation of HbA1c level with the SYNTAX score and GRACE score. Results of the accuracy-test were statistically significant at *α* = 0.05, *P* < 0.05.

The article "The Level of HbA1c Evaluates the Extent of Coronary Atherosclerosis Lesions and the Prognosis in Diabetes with Acute Coronary Syndrome" was retracted in 2023. Reason: concerns about the peer review.

## 3. Results

### 3.1. Baseline Patient Characteristics

Between January 2019 and December 2020, there was a total of 233 patients (power analysis and sample size: group sample sizes of 81 and 81 achieve 90.036% power to reject the null hypothesis of equal means when the population mean difference is *μ*1 − *μ*2 = 23.9 − 26.8 = −2.9 with standard deviations of 4.8 for group 1 and 6.2 for group 2 and with a significance level (alpha) of 0.050 using a two-sided two-sample unequal-variance *t*-test). Considering the loss to follow-up rate of 10%, at least 89 patients are needed in each of the two groups, and a total of at least 178 patients will be included) having diabetes complicated with ACS were enrolled and assigned to two groups according to the level of HbA1c: HbA1c ≤ 7%group (*n* = 92) and HbA1c > 7%group (*n* = 141).

Table 1 shows the clinical characteristics of the participants in the two groups. There were no statistically significant differences between the two groups (*p* > 0.05) except in previous PCI, fasting blood glucose, TG, and LDL-C (*p* < 0.05).

### 3.2. Comparison of Different Types of ACS in the Two Groups

Table 2 compares the incidence of the ACS types between the two groups. The proportion of STEMI was higher in the HbA1c ≤ 7%group (*p* < 0.05), and the proportion of NSTEMI was higher in the HbA1c > 7%group, but this was not statistically significant (*p* > 0.05). There were no statistically significant differences in UA between the two groups (*p* > 0.05).

### 3.3. Comparison of the SYNTAX Score, GRACE Score, LVEDV, and LVEF in the Two Groups

Table 3 shows that the SYNTAX score and GRACE score were both higher in the HbA1c>7% group (27.19 ± 6.17 vs. 24.33 ± 5.00*p* < 0.001 and 114.84 ± 23.95 vs. 105.38 ± 19.03*p* = 0.002, respectively). There were no statistically significant differences in LVEDV or LVEF between the two groups (*p* > 0.05).

### 3.4. Correlation of HbA1c Level with the SYNTAX Score and GRACE Score

In Figures 1 and 2, the linear regression analysis shows that there was a significant positive correlation of HbA1c level with GRACE score (*r* = 0.156, *F* = 5.784, *p* = 0.017, *n* = 233) and SYNTAX score (*r* = 0.237, *F* = 13.788, *p* = 0.000581, *n* = 233).

### 3.5. Comparison of MACEs in the Hospital and 12 Months after Discharge in the Two Groups

Table 4 shows the MACEs in the hospital. In the HbA1c ≤ 7%group, this included one patient who needed target lesion revascularization and two patients who suffered ventricular tachycardia/fibrillation. In the HbA1c > 7%group, two patients experienced recurrent ACS, three patients experienced ventricular tachycardia/fibrillation, two patients needed target lesion revascularization, and two patients died. The total MACEs rate showed no significant difference between the two groups (*p* > 0.05).

The article "The Level of HbA1c Evaluates the Extent of Coronary Atherosclerosis Lesions and the Prognosis in Diabetes with Acute Coronary Syndrome" was retracted in 2023. Reason: concerns about the peer review.

MACEs at 12 months after discharge: In the HbA1c ≤ 7%group, two patients needed target lesion revascularization, and one patient experienced recurrent ACS, while in the HbA1c > 7%group, five patients experienced recurrent ACS, seven patients needed target lesion revascularization, and three patients died. The total MACEs rate was significantly different between the two groups (*p* < 0.05).

## 4. Discussion

As one of the advanced glycation end products, the level of HbA1c can reflect the blood glucose control level of diabetic patients over a prolonged period. This study also suggested that the level of fasting blood glucose in the HbA1c>7% group was significantly higher than that in the HbA1c ≤7% group.

HbA1c level can be used as a prognostic indicator for other diseases in diabetic and nondiabetic patients. A higher HbA1c level in patients undergoing coronary angiography is associated with an increased prevalence of comorbidities [8]. Higher HbA1c level is associated with higher coronary and peripheral atherosclerotic burden in nondiabetic patients [9].

A previous study has shown that HbA1c testing offers a simple and effective way to screen for diabetes with ACS [12]. In the context of diabetes, a significant number of patients with STEMI may not have serious coronary artery stenosis, which is mainly caused by acute thrombosis resulting from unstable plaque rupture; however, NSTEMI patients often have poor long-term glycemic control, which results in a sustained increase in HbA1c levels. As a glycosylation end product, HbA1c causes dysfunction of vascular endothelial cells, decreases endogenous fibrinolysis activity, enhances platelet agglutination, increases plasma plasminogen, quickens smooth muscle proliferation and extracellular matrix deposition, accelerates age-related endothelial dysfunction, and finally leads to a higher incidence of NSTEMI [13–18]. Moreover, the results of this study indicate that fasting blood glucose, TG, and LDL-C were higher in the HbA1c > 7%group.

Another study has shown that HbA1c level can be used as an independent marker to determine the probability and severity of CAD in nondiabetic individuals and as a useful marker in primary care to predict CAD [19]. In diabetes patients, Ravipati found that the higher the HbA1c level was, the more coronary artery lesions were found on coronary angiography [20]. However, they ignored the location, occlusion, calcification, bifurcation, and diffusion of coronary artery disease; so, it was not possible to objectively evaluate its severity. The results of our study suggest that the incidence of STEMI is higher in patients with HbA1c ≤ 7%, while the incidence of NSTEMI is higher in patients with HbA1c > 7%. In this study, the SYNTAX score, which is an assessment of CAD based on coronary artery anatomy [10], was used as the evaluation index of coronary disease, thus increasing the objectivity of our results. Studies have shown that there is a significant correlation between HbA1c level and CHD severity as measured by the SYNTAX score [21].

The article "The Level of HbA1c Evaluates the Extent of Coronary Atherosclerosis Lesions and the Prognosis in Diabetes with Acute Coronary Syndrome" was retracted in 2023. Reason: concerns about the peer review.

The results of our study showed that the higher the level of HbA1c, the higher the SYNTAX score in diabetes with ACS. The possible mechanism is that HbA1c, as an advanced glycation end product, promotes the occurrence and progression of coronary atherosclerosis [13–18]. Hyperglycemia and high LDL-C are known to be the main risk factors for CHD. Long-term hyperglycemia and high LDL-C cause an inflammatory response and oxidative stress, which contribute to the development of coronary artery atherosclerosis.

Therefore, it is of great significance to delay or prevent atherosclerosis and the development of cardiovascular diseases by strictly controlling blood glucose, reducing HbA1c and improving the function of vascular endothelial cells, thus preventing the progression of coronary atherosclerosis.

The relationship between HbA1c level and the prognosis of CHD is still controversial. HbA1c variability is an independent predictor of the incidence of poststent restenosis in diabetes [22]. HbA1c provides significant prognostic information in CAD [23]. HbA1c level has been shown to be a predictor of mortality and major adverse events in patients with NSTEACS, rather than the admission glucose level or the fasting glucose level [24]. The observed U-shaped relationship indicates that both high and low HbA1c levels might be associated with all-cause mortality [25].

However, other studies have shown that HbA1c level is not associated with short-term cardiovascular outcomes in patients with diabetes complicated with ACS [26]. The GRACE score has been used to evaluate the prognosis of patients with ACS and assess the risk of recurrent myocardial infarction or death during and after hospitalization, general increases using evidence-based therapies for ACS were observed in the expanded GRACE [27]. The results of this study suggest that with the increase in HbA1c level, the GRACE score also gradually increases, indicating that higher HbA1c brings a worse prognosis in diabetes patients with ACS. The possible mechanism is that in patients with higher HbA1c levels due to long-term hyperglycemia, higher LDL-C levels and associated diseases lead to severe coronary atherosclerotic lesions, which are often combined with cardiac and renal insufficiency, eventually leading to the poor general condition and poor prognosis.

The article "The Level of HbA1c Evaluates the Extent of Coronary Atherosclerosis Lesions and the Prognosis in Diabetes with Acute Coronary Syndrome" was retracted in 2023. Reason: concerns about the peer review.

In our study, death, ventricular tachycardia/fibrillation, recurrent myocardial infarction and target lesion revascularization were the definition of MACEs. The results of this study suggested that there was a positive correlation between HbA1c level and the total MACEs rate 12 months after discharge in diabetic patients with ACS. This link may be related to severe coronary artery disease, high GRACE score, various complications of diabetes and long-term hyperglycemia itself [28].

## 5. Conclusion

However, the results of this study showed that regardless of the HbA1c level, there was no significant difference in LVEDV or LVEF between the two HbA1c groups. We used to think that higher HbA1c levels were associated with more severe coronary artery disease, more severe myocardial ischemia, and more severe myocardial cell damage or apoptosis, leading to cardiac hypertrophy and decreased LVEF. However, the results of this study go against that; so, further research is needed to explain this discrepancy.

In conclusion, this study showed that the level of HbA1c was positively correlated with the SYNTAX score, GRACE score, and total MACEs at 12 months after discharge in diabetes patients with ACS. The higher the HbA1c level, the more severe the coronary atherosclerotic lesion and the worse the prognosis in diabetes with ACS.

This study has several limitations. First, this was a single-center study with a relatively small sample size. Second, the follow-up was short, and patients had only one hospitalization period; so, the change in HbA1c level and its correlation with clinical events could not be evaluated. The results of this study need to be confirmed by large, multicenter, long-term follow-up studies implementing evidence-based medicine.

Our results indicate that HbA1c level is positively correlated with the extent of coronary atherosclerotic lesions and the prognosis in diabetes with ACS. The higher the HbA1c level is, the more severe the coronary atherosclerotic lesion and the worse the prognosis in diabetes with ACS will be. The data analyzed in this study are available, and any access needs to preserve the privacy of patients and researchers.

## Figures and Tables

**Figure 1:** Correlation of HbA1c level with the SYNTAX score.

The article "The Level of HbA1c Evaluates the Extent of Coronary Atherosclerosis Lesions and the Prognosis in Diabetes with Acute Coronary Syndrome" was retracted in 2023. Reason: concerns about the peer review.

**Figure 2:** Correlation of HbA1c level with the GRACE score.

**Table 1:** Comparison of the general clinical data of the participants in the two groups.

Group	HbA1c ≤ 7%group (*n* = 92)	HbA1c > 7%group (*n* = 141)	*t*/*χ*^2^	*p*
Age (years)	62.82 ± 12.093	64.03 ± 12.669	0.727	0.468
Male *n* (%)	68 (73.91)	98 (69.50)	0.528	0.467
Hypertension *n* (%)	43 (46.74)	68 (48.22)	0.049	0.824
Cerebrovascular accident n (%)	31 (33.70)	57 (40.43)	1.073	0.300
Smoking history *n* (%)	23 (25.00)	43 (30.50)	0.828	0.363
BMI	24.6 ± 7.23	26.8 ± 8.71	0.481	0.397
Previous PCI *n* (%)	6 (6.52)	24 (17.02)	5.471	0.019
Previous ACS *n* (%)	4 (4.35)	13 (9.22)	1.300	0.254
Fasting blood glucose (mmol/L)	6.26 ± 1.393	8.74 ± 3.757	6.080	<0.01
TG (mmol/L)	1.60 ± 1.156	2.11 ± 1.846	2.347	0.020
TC (mmol/L)	4.30 ± 01.297	4.23 ± 1.195	0.383	0.702
LDL-C (mmol/L)	2.64 ± 1.062	2.32 ± 1.109	2.171	0.031
HDL-C (mmol/L)	1.11 ± 0.422	1.03 ± 0.261	1.805	0.072

BMI: body mass index; PCI: percutaneous coronary intervention; ACS: acute coronary syndrome; TG: triglyceride; TC: total cholesterol; LDL-C: low-density lipoprotein cholesterol; HDL-C: high-density lipoprotein cholesterol.

**Table 2:** Comparison of incidence of the ACS types in two groups *n* (%).

Group	UA *n* (%)	NSTEMI *n* (%)	STEMI *n* (%)
HbA1c ≤ 7% (*n* = 92)	45(48.91)	20 (21.74)	27 (29.35)
HbA1c > 7% (*n* = 141)	73 (51.77)	47 (33.33)	21 (14.90)
*χ* ^2^	1.182	3.653	7.111
*p*	0.670	0.056	0.008

UA: unstable angina pectoris; NSTEMI: non-ST-segment-elevation myocardial infarction; STEMI: ST-segment-elevation myocardial infarction.

**Table 3:** Comparison of the SYNTAX score, GRACE score, LVEDV, and LVEF in the two groups.

Group	SYNTAX score	GRACE score	LVEDV (mm)	LVEF (%)
HbA1c ≤ 7% (*n* = 92)	24.33 ± 5.00	105.38 ± 19.03	52.27 ± 5.15	59.53 ± 10.27
HbA1c > 7% (*n* = 141)	27.19 ± 6.17	114.84 ± 23.95	52.09 ± 5.38	59.68 ± 9.79
*t*	3.724	3.189	0.253	0.111
*p*	<0.01	0.002	0.800	0.912

GRACE: The Global Registry of Acute Coronary Events score; LVEF: left ventricular function; LVEDV: left ventricular end-diastolic volume; MACE: major adverse cardiovascular events.

**(a):** 

	HbA1c ≤ 7%(*n* = 92)	HbA1c > 7% (*n* = 141)	**x** ^2^	*p*
In-hospital clinical outcome				
Recurrent ACS, *n*	0	2	—	—
Target lesion revascularization, *n*	1	2	—	—
Ventricular tachycardia/fibrillation, *n*	2	3	—	—
Death, n	0	2	—	—
Total major adverse cardiac events, *n*	3	9	0.564	0.453

**(b):** 

	HbA1c ≤ 7% (*n* = 92)	HbA1c > 7% (*n* = 139)	*x* ^2^	*p*
Clinical outcomes 12 months after discharge				
Recurrent ACS, *n*	1	5	—	—
Target lesion revascularization, *n*	2	7	—	—
Death, *n*	0	3	—	—
Total major adverse cardiac events, *n*	3	15	4.128	0.022

Death, recurrent ACS, ventricular tachycardia/fibrillation, and target lesion revascularization were defined as the major adverse cardiac events.

The article "The Level of HbA1c Evaluates the Extent of Coronary Atherosclerosis Lesions and the Prognosis in Diabetes with Acute Coronary Syndrome" was retracted in 2023. Reason: concerns about the peer review.

## Data Availability

The data and materials used and/or analyzed in this study are available from the corresponding author on reasonable request.

## Abbreviations

ACS: Acute coronary syndrome
GRACE: The global registry of acute coronary events
LVEF: Left ventricular function
LVEDV: Left ventricular end-diastolic volume
MACEs: Major adverse cardiac events
IDF: The international diabetes federation
CVDs: Cardiovascular diseases
CAD: Coronary artery disease
UA: Unstable angina pectoris
NSTEMI: Non-ST-segment-elevation myocardial infarction
STEMI: ST-segment-elevation myocardial infarction
BMI: Body mass index
PCI: Percutaneous coronary intervention
TG: Triglyceride
TC: Total cholesterol
LDL-C: Low-density lipoprotein cholesterol
HDL-C: High-density lipoprotein cholesterol.
